RETRACTED

# Safety and Efficacy of Tirofiban Combined with Statins in the Perioperative Period of Intracranial Aneurysms: Systematic Review and Meta-Analysis

**DOI:** 10.1155/2022/8264261

**Published:** 2022-09-30

**Authors:** Ming Hao, Rui Liu, Feiping Yan, Youcai Luo

**Affiliations:** ^1^Department of Neurosurgery, The Second Hospital of Yulin, Yilin City Shaanxi Province 719000, China; ^2^Department of Neurology, The First Hospital of Yulin, Shaanxi Province 719000, China; ^3^Department of Neurosurgery, The First Hospital of Yulin, Shaanxi Province 719000, China

## Abstract

**Objective:**

In order to verify the safety and effectiveness of tirofiban combined with statins in the perioperative period of intracranial aneurysms, this study adopts systematic review and meta-analysis, so as to comprehensively understand the situation of intracranial aneurysms in the perioperative period, and tirofiban combined with statins was finally determined as an effective treatment drug.

**Methods:**

This study used systematic retrospective analysis and selected 80 patients with intracranial aneurysms treated in our hospital from June 2021 to June 2022 as the research objects. Through conventional drugs and tirofiban combined with statins used in this study, the intracranial levels, the probability of aneurysm rupture, and postoperative complications of the two groups were observed and recorded.

**Results:**

The analysis of 80 patients with intracranial aneurysms showed that the influence of intracranial levels in the observation group was better than that in the reference group, the rupture of aneurysms in the observation group was lower than that in the reference group, and the incidence of postoperative complications in the observation group was lower than that in the reference group.

**Conclusion:**

Through simulation verification, it is concluded that tirofiban combined with statins is safe and effective in the perioperative application of intracranial aneurysms. This drug can improve vascular recanalization, reduce the incidence of cerebrovascular disease events, and reduce the incidence of rebleeding. Its therapeutic effect is worthy of wide clinical application and promotion.

## 1. Introduction

Intracranial aneurysms are tumor like protrusions caused by abnormal changes in local blood vessels of the intracranial cerebral artery wall, resulting in local vascular wall damage. Under the action of hemodynamic load and other related factors, they gradually expand and form abnormal protrusions. Aneurysm is a kind of cerebrovascular disease, which is very likely to have rupture and bleeding. Once rupture and bleeding occur, it will have a great impact on health, and there will be sequelae of nerve loss. When the amount of bleeding is large, it is easy to cause death. Tirofiban, as a more powerful antiplatelet drug, has an effect on platelet aggregation induced by various factors. It can inhibit platelet aggregation by inhibiting fibrinogen and platelet synthesis-related receptors, so as to prolong the time of bleeding, inhibit thrombosis, or reduce the size of thrombosis. Tirofiban, as a representative inhibitor, is used in the treatment of intracranial aneurysm vascular embolism. This drug can not only be used for remedial treatment after thrombosis but also play a preventive role. Statins can effectively reduce the level of blood lipids; reduce the inflammatory response of vascular endothelial cells; regulate vascular endothelium, anti-inflammatory, and antioxidant; improve vascular reactivity; and play a positive role in reducing the incidence of cerebrovascular disease events. Statins can limit the occurrence and development of intracranial aneurysms and effectively reduce the risk of aneurysm rupture. Tirofiban combined with statins provides a new treatment method and direction for intracranial aneurysms and has a great application prospect in perioperative treatment. Xiaojuan and Danfeng [1] discussed the effect of perioperative nursing combined with hyperbaric oxygen therapy in patients with intracranial aneurysms, which can effectively reduce the incidence of complications in patients with intracranial aneurysms, highlighting the importance of perioperative nursing. Di et al. [2] systematically evaluated the safety and effectiveness of tirofiban in the perioperative period of intracranial aneurysms, which can significantly reduce the occurrence of thromboembolic events and intracranial hemorrhage events. Therefore, they believed that the use of tirofiban antiplatelet therapy in the perioperative period is safe and effective and can provide evidence-based reference for clinical rational drug use. Weidong et al. [3] analyzed retrospectively the clinical data of perioperative patients with intracranial aneurysms in neurosurgery, evaluated the therapeutic effect of tirofiban in the perioperative period, and concluded that tirofiban is a safe and effective treatment for this disease by recording and analyzing the successful thrombolysis rate, intracranial hemorrhage, and discharge prognosis of patients after surgery. Gang et al. [4] summarized the perioperative complications of intravascular embolization for intracranial aneurysms, analyzed the high-risk related factors affecting the occurrence of complications, and retrospectively analyzed the patient's case data. Multivariate logistic regression showed that ischemia and hemorrhage were the perioperative complications of this disease, with a high risk of occurrence. Jian et al. [5] analyzed the clinical significance of the morphological and hemodynamic characteristics of the disease in predicting the risk of rupture and compared the morphological parameters and hemodynamic parameters of aneurysms, which is helpful to evaluate the risk of rupture. Binghao et al. [6] pointed out that the disease is a disease with a high mortality and disability rate among cerebrovascular diseases. Once aneurysmal hemorrhage occurs, it is extremely critical. The urgent task is to conduct rupture risk assessment, obtain morphological indicators of intracranial aneurysms, and deal with aneurysms with high rupture risk [6]. Gang [7] discussed that statins can effectively reduce the risk of cardiovascular disease, and the clinical guidelines recommend statins as the first-line treatment to prevent cardiovascular disease. This study is a cerebrovascular disease. Statins combined with other drugs can also effectively reduce the risk. Lin [8] retrospectively analyzed the compliance status and related factors of statins in secondary prevention of ischemic cerebrovascular disease and analyzed the risk of ischemic cerebrovascular disease with multiple correspondences. Jiali [9] systematically evaluated and meta analyzed the therapeutic effect of statins on aneurysmal hemorrhage. When the disease ruptures, blood flows into and accumulates in the subarachnoid space, causing a clinical syndrome, which is a common and very serious disease [9]. Zhouqin and Chunhua [10] collected the clinical research literature of patients with intracranial aneurysms, performed meta-analysis on the relevant literature that met the requirements, and systematically reviewed and evaluated the incidence of postoperative adverse reactions of patients. Kim (2022) et al. summarize the treatment effect and safety of patients when summarizing the thermal ablation treatment of intrahepatic cholangiocarcinoma [11], which can provide reference value for this study. Jie et al. [12] discussed the safety and effectiveness of intravenous tirofiban after intravascular treatment of acute cerebral infarction. Tirofiban can improve the discharge score of patients with intravascular. It has been proved that intravenous tirofiban is safe. Fuxing et al. [13] discussed the safety and effectiveness of aspirin in the treatment of ischemic cerebrovascular diseases. It has been proved that it can improve indicators and have significant treatment effect and high safety. In this study, aspirin was used as the conventional drug in the reference group to analyze the safety and effectiveness of other drugs in the treatment of cerebrovascular diseases. In this study, the general data of patients were systematically reviewed by multivariate logistic regression; from the statistical results, the feasibility and safety of tirofiban in treatment have been confirmed, which can reduce the incidence of bleeding. Combined with statins in the treatment of intracranial aneurysms during perioperative period, the activity of inhibitory factors can inhibit the development of aneurysms and further reduce the incidence of cerebrovascular disease events.

RETRACTED

## 2. Meta-Analysis of Intracranial Aneurysms

### 2.1. Clinical Application of Tirofiban Combined with Statins

Tirofiban as a nonpeptide high selective antagonist can inhibit platelet aggregation and adhesion most rapidly, directly, and completely and can effectively prevent the binding of fibrinogen and receptor. Statins can effectively reduce the blood lipid level of patients and reduce the inflammatory reaction of vascular endothelial cells. Statins are not only aimed at cardiovascular diseases but also benefit the blood vessels of the whole body. They can reduce sclerotic plaque and prevent thrombosis. They can play an obvious therapeutic effect in the treatment of cerebrovascular diseases and have high safety.

### 2.2. Clinical Application of Conventional Drugs

The reference group of this study was treated with conventional drugs such as aspirin and nimodipine. Aspirin is an anticoagulant. For the thrombotic pathway, it can inhibit one or more of the many conduction pathways leading to platelet aggregation, so as to inhibit platelet aggregation and avoid the occurrence of thrombosis caused by platelet aggregation. Nimodipine is used to improve blood circulation and prevent and treat ischemic nerve injury caused by aneurysms. The drug has a good effect on patients with vascular dementia.

### 2.3. Meta-Analysis of Drugs for Intracranial Aneurysms

In this study, meta-analysis was used to compare and synthesize the discussion of tirofiban combined with statins in the perioperative period of intracranial aneurysms. According to the statistical method of the research results of the problems related to the topic, relevant studies were comprehensively collected through retrieval and strictly evaluated and analyzed one by one, and those that did not conform to the topics related to tirofiban combined statins and intracranial aneurysms, as well as the repeated publication of tirofiban combined statins. The relevant literature of intracranial aneurysms, after systematic detection, evaluation, and summary, and quantitative combined analysis in the systematic review, is helpful to explore the consistency and other differences of the therapeutic effect of tirofiban combined with statins in the treatment of intracranial aneurysms. Rigorous meta-analysis can make a more objective evaluation. The clinical similarity and methodological similarity of the included studies are good. The results of tirofiban combined with statins in the perioperative period of intracranial aneurysms in this study finally proved to be safe and effective. It has super high reliability.

RETRACTED

## 3. General Information and Methods

### 3.1. General Information of Patients

This study adopts systematic retrospective analysis and selects 80 patients with intracranial aneurysms treated in our hospital from June 2021 to June 2022 as the research object. The patients are divided into two groups according to odd and even grouping, with 40 patients in each group. Among them, 40 patients treated with conventional drugs, such as aspirin and nimodipine, were used as the reference group, including 15 male patients and 25 female patients. The age range was 40 to 75 years old, and the median age was (55.4 ± 3.8) years old; 40 patients treated with tirofiban combined with statins were used as the observation group, including 13 male patients and 27 female patients. The age range was 42 to 73 years old, and the median age was (54.1 ± 3.7) years old. After univariate *t*-test, the general data of the two groups were not statistically significant (*p* > 0.05), which was comparable.

### 3.2. Case Selection and Exclusion

#### 3.2.1. Case Inclusion Criteria

1. The patient and his family members have given their informed consent and signed the informed consent form
2. No Alzheimer's disease or other cognitive impairment, clear consciousness, and certain expression ability
3. There were no other serious complications

#### 3.2.2. Case Exclusion Criteria

1. Noncompliant patients
2. Have acute and chronic infectious diseases
3. Patients with a variety of basic diseases

### 3.3. Observation Index

1. Observe and record the influence of intracranial levels in the two groups
2. The probability of aneurysm rupture was observed and recorded in the two groups
3. The postoperative complications of the two groups were observed and recorded

## 4. Method

### 4.1. Perioperative Methods

Before the perioperative period, the patients were given psychological intervention to relieve the tension of the patients, explain the disease knowledge to the patients, reduce the pressure and tension of the patients, enhance the confidence of the patients, and receive treatment with the best psychological state.

After the operation of intracranial aneurysms, the patients in the reference group were treated with aspirin and nimodipine, the changes of vital signs were monitored, and the changes of the patient's condition were recorded. After the operation, the patients were asked to take an absolute lying position, and the patients were asked to relax their heads, do not use force, and do not shake their heads. Let patients have a good rest, ensure adequate nutrition and sleep, reduce intracranial pressure, pay attention to posture, and prevent rebleeding. The observation group used tirofiban combined with statins to ensure vascular recanalization. Observe and ask the patient's condition changes in time during the treatment. Observe the clinical symptoms and adverse reactions of patients after medication. The effect of a reasonable safe dose of medication on a high dose will lead to aneurysm rupture. Monitor the ECG, blood vessel level, and vital signs of patients; and deal with them in time once abnormalities are found. Strictly follow the doctor's advice on medication. If the patient is found to have a slight headache, or accompanied by nausea, vomiting, and other conditions, it should be reported to the surgeon in time to check whether the patient has increased intracranial pressure.

RETRACTED

Eat more crude fiber food, digestible food, and drink more water after operation. Drink water slowly to prevent choking reaction. Pay attention to rest, and avoid fatigue and emotional excitement. After the operation, take drugs strictly according to the doctor's advice to improve the patient's medication compliance.

### 4.2. Statistical Methods

The systematic review of clinical data was studied by meta-analysis using IBM SPSS 24.0 data analysis platform and Revman 5.3 software. Observe the law of data distribution, use Spearman correlation analysis method to discuss the correlation of data, and use curve estimation and linear regression analysis to observe the statistical law of data. In all analyses, the significance *p* value of statistical data is considered to be in the confidence space when *p* < 0.05, and the statistical result is considered to be in the absolute confidence space when *p* < 0.01.

## 5. Simulation Verification

### 5.1. Compare the Effects of the Two Methods on Intracranial Levels

After the occurrence of intracranial aneurysms, they often develop further, leading to the expansion of aneurysms, which seriously causes the injury and dysfunction of intracranial arterial endothelial cells. When drugs are used, it will have a direct impact on the diameter of aneurysm. Collagen fiber is an important part of extracellular matrix. Changes in collagen fiber synthesis will lead to changes in the thickness of aneurysm wall. Aneurysmal inflammatory factors such as TNF-*α*, after activation, will cause intracranial inflammatory reaction. After drug treatment, it can inhibit the spread of inflammation and hinder the development of aneurysms.

RETRACTED

At this stage, the relationship between aneurysm diameter, aneurysm wall thickness, and TNF was observed-*α*. The influence of intracranial level is made into Table 1 as follows.

Table 1 shows the comparison results of the two groups of data. The diameter of the aneurysm in the observation group is about 3.87 cm and that in the control group is about 4.78 cm, which is significantly smaller than that in the control group. In addition, the thickness of the aneurysm in the control group is thinner than that in the observation group, inflammatory factor TNF in control group- *α* More than observation group. There was a statistical relationship between *t* < 10.000 and *p* < 0.05. Through visual analysis of the above data, Figures 1 and 2 are obtained.

As shown in Figures 1 and 2, the diameter, thickness, and TNF of intracranial aneurysms in the two groups are shown-*α*. According to two sets of TNF- *α*The results of the level comparison can be seen intuitively that tirofiban combined with statins has a better therapeutic effect than conventional drugs. There is a wide gap between the two groups. This drug combined with statins can reduce inflammatory factors and improve the progress of aneurysm. All levels of intracranial are better than those of conventional drugs. It can be indirectly concluded that tirofiban combined with statins can effectively eliminate inflammation and inhibit the development of intracranial aneurysms.

### 5.2. Two Methods for Aneurysm Rupture

The incidence of thromboembolism in intracranial aneurysm surgery is high. Embolizing intracranial aneurysms has certain risks, and aneurysms are very fragile, so, in order to prevent and treat thromboembolism, drug intervention is needed. However, after drug intervention, platelet function will be abnormal, increasing the risk of aneurysm rupture. Tirofiban combined with statins can effectively improve the rupture of aneurysms.

Now, we study the probability of aneurysm rupture under the two methods; analyze the probability of intracranial hemorrhage, subarachnoid hemorrhage, and head pain after rupture; and make Table 2.

As shown in Table 2, the probabilities of intracranial hemorrhage, subarachnoid hemorrhage, and head pain in the observation group were 2.5%, 3.75%, and 5%, respectively, while the probabilities of the control group were 13.75%, 18.75%, and 16.25%, respectively. There is a result of *T* < 10.000 and *p* < 0.05 between the two comparisons of the data, that is, there is a statistical difference between the data, which can be considered that different drugs have a certain impact on the rupture of aneurysms. According to the above data, Table 2 is made into a visual diagram as follows.

RETRACTED

Tirofiban has a short half-life, and the recovery rate of platelet function is higher after the withdrawal of combined statins. According to the analysis of Figure 3, the use of tirofiban combined with statins has a small risk of aneurysm rupture, and the probability of adverse events after rupture is low. It can be considered that tirofiban combined with statins is safer than conventional drugs.

### 5.3. Comparison of Postoperative Complications

For intracranial aneurysms, surgery should be actively used to maintain normal blood flow. There may be a series of complications after operation, such as hydrocephalus, new cerebral infarction, or recurrent aneurysm, so drugs should be used after operation to improve the prognosis. Now compare the incidence of postoperative complications between the two groups, study and analyze the prognosis of the two groups, and make the data into Table 3.

In order to better analyze the incidence of postoperative complications in the two groups, the following Figure 4 is obtained by visualizing the data in Table 3.

Complications are the main problem after aneurysm surgery. In Table 3 and Figure 4, only one person in the observation group has a new cerebral infarction after surgery, with a probability of 1.25%, while the probability of the control group is 13.78%. The probability of complications in the observation group was significantly lower than that in the control group, and the prognosis was good. Based on the above data, it can be concluded that tirofiban combined with statins is more effective and safe in the prognosis of intracranial aneurysm surgery.

## 6. Summary

This study focused on the observation and analysis of the safety and effectiveness of tirofiban combined with statins in the perioperative period of intracranial aneurysms. Through statistical methods and meta-analysis, logistic regression method for systematic review and the influence data of intracranial levels in the observation group were significantly better than those in the reference group, and the aneurysm rupture rate and postoperative complication rate in the observation group were also lower than those in the reference group. It can be concluded that tirofiban combined with statins can improve vascular endothelial function, protect nerves, and resist thrombosis. It has been proved that intravenous tirofiban combined with statins is safe and effective in the perioperative period of patients with intracranial aneurysms. Tirofiban combined with statins has an exciting prospect in the treatment of intracranial aneurysms, which can provide a good basis for subsequent treatment. To sum up, tirofiban combined with statins has an important impact on its clinical effect and has the significance of clinical treatment promotion.

RETRACTED

## Figures and Tables

**Figure 1:** Comparison of aneurysm diameter and aneurysm wall thickness between the two groups.

**Figure 2:** Two groups of TNF-*α* horizontal comparison chart.

**Figure 3:** Comparison of aneurysm rupture.

**Figure 4:** Comparison of postoperative complication rate.

**Table 1:** Changes of intracranial levels.

Group	Aneurysm diameter (cm)	Aneurysm wall thickness (*μ*m)	TNF-*α* (ng/l)
Observation group	3.87 ± 0.23	0.78 ± 0.15	35.07 ± 3.75
Control group	4.78 ± 0.25	0.56 ± 0.13	89.73 ± 4.38
*t*	8.572	9.134	8.264
*p*	0.01	0.013	0.018

**Table 2:** Comparison of aneurysm rupture.

Group	Intracranial hemorrhage (%)	Subarachnoid hemorrhage (%)	Head pain (%)
Observation group	2.5	3.75	5
Control group	13.75	18.75	16.25
*t*	8.453	8.612	7.685
*p*	0.015	0.009	0.02

**Table 3:** Comparison of postoperative complications.

Group	Hydrocephalus (%)	New cerebral infarction (%)	Recurrent aneurysm (%)
Observation group	3.75	1.25	6.25
Control group	10	13.75	16.25

## Data Availability

The data underlying the results presented in the study are available within the manuscript.
